# Compound Shuganjieyu Capsule on CYP450 Enzyme Activity

This article has been retracted.

**DOI:** 10.1155/2022/3228738

**Published:** 2022-10-13

**Authors:** Yunqiu Tang, Yunxia Li

**Affiliations:** ^1^The Third People Hospital of Chengdu, Chengdu, Sichuan Province, 610506, China; ^2^School of Pharmacy, Chengdu University of Traditional Chinese Medicine, Chengdu, Sichuan Province, 610506, China

## Abstract

**Objective:**

To evaluate the potential drug-drug interactions of the Shuganjieyu capsule by establishing a Chronic Unpredictable Mild Stress (CUMS) depression model combined with the Cocktail probe substrate method.

**Methods:**

The whole study was divided into the single-dose and multiple-dose groups. Animals were randomly divided into further subgroups in each group. Following chronic unpredictable mild stress model development, Shuganjieyu capsules were administered to the drug administration group. The single-dose subgroup received the drug for one day, and the multiple-dose subgroup received the drug for three months. Liver microsomes of each group were extracted, and the effects of the Shuganjieyu capsule on the CYP450 enzyme were investigated by liquid chromatography-mass spectrometry (LC-MS) (LC-MS) based on the Cocktail probe substrate method. The immunohistochemical method and RT-qPCR were used to detect the activity of CYP450 immunoprotein in rat liver.

**Results:**

In the single-dose subgroup, there were no statistical differences between the administration and model groups. In the multiple-dose subgroup, the conversion and protein expression rates of CYP1A2 and CYP2C19 were significantly increased in the model group compared with the blank group. In the administration group, the conversion and protein expression rates of CYP1A2 and CYP2C19 were inhibited.

**Conclusion:**

Long-term administration of the Shuganjieyu capsule could relieve depression-related behaviors in CUMS rats and downregulate the CYP1A2 and CYP2C19 enzyme activities in CUMS rats by inhibiting the expression of CYP1A2 and CYP2C19 protein. Long-term administration of the Shuganjieyu capsule may affect the bioavailability of other drugs metabolized by CYP1A2 and CYP2C19 enzymes, but the clinical guidance's specific significance needs to be clarified further.

## 1. Introduction

Cytochrome P450 (CYP450) is a super large gene family composed of a variety of isoenzymes involved in more than 90% of the body's drug metabolism [1, 2]. CYP1, CYP2, and CYP3 gene families are the leading CYP families involved in the metabolism of most drugs in the body. Cytochrome P450 enzymes are abundant in the liver. CYP1A2, CYP2C9, CYP2C19, CYP2D6, CYP3A4, and CYP3A5 participate in most drug metabolism. The increase or decrease of their activity is likely to lead to drug-drug interaction [3, 4], change the bioavailability of drugs in the body, affect the therapeutic effect of drugs, and even lead to toxic and side effects. Therefore, the research on P450 enzymes plays a vital role in studying drug metabolism. The cocktail probe substrate method refers to various relatively low doses of probe drugs given simultaneously. The metabolic rate or other metabolic typing indicators of each probe drug in biological samples are measured by ultra-high-performance liquid chromatography-mass spectrometry (LC-MS) (UPLC-MS/MS) to obtain the phenotypic information of multiple metabolic enzymes, which is of great significance for the dose design of those with multiple metabolic pathways [5]. The main components of the Shuganjieyu capsule are Hypericum perforatum and acanthopanax senticosus. Its functions contain soothing the liver, relieving depression, and calming the mind to improve the symptoms of depression [6]. This study was aimed at investigating the enzyme inhibition or induction capability of Shuganjieyu capsules in animals to elucidate the potential for drug-drug interactions by estimating liver enzyme levels by employing analytical techniques like LCMS and UHPLC-MS/MS.

## 2. Materials and Methods

The following are used in the study: testosterone, paracetamol, phenacetin, and NADPH (Beijing Solarbio Science & Technology Co., Ltd. China); dextran, dextromethorphan, omeprazole, 5-hydroxy omeprazole, tolbutamide, 4-hydroxytolbutamide, and 6*β*-hydroxytestosterone (Toronto Research Chemicals); BCA protein Kit (Lianke Biotechnology Corporate Limited, No. a81911151); primer (synthesized by Tsingke Biotechnology Co., Ltd.); reverse transcription Kit (Tsingke Biotechnology Co., Ltd., No. 20190328); and CYP1A2, cyp2d1, CYP3A4, CYP3A1, CYP2C19, and CYP2C11 antibodies (Abcam Company).

### 2.1. Instrument

The following are used in the study: UPLC-high-resolution time-of-flight mass spectrometer (including quaternary gradient pump autosampler two-stage tube array detector column temperature chamber), ACQUITY (Synaptic G2, Waters Corporation of the United States); Liquid transfer gun (Dragon, KE0003087/KA0056573); Histochemical pen (Gene tech, GT1001); BS 124 S-type analytical balance (Beijing sartorius Instruments Co., Ltd.); Alleger X-12 centrifuge (BECKMAN Coulter, USA); Varioskan flash-3001 microplate reader (Thermo Scientific, USA); and QTOWER real-time fluorescent quantitative PCR instrument (ANALYTIKJENA, Germany).

### 2.2. Experimental Grouping

Healthy male Sprague Dawley rats (weight = 200 ± 10 g) were purchased from Chengdu Gossy Experimental Animals Co. Ltd., China, and were acclimatized for seven days with free access to food and water. The animals were randomly first divided into the single administration and long-term administration groups. The single administration group animals were further divided into the blank control group, model group, and administration group (who were administered doses at rates of 65 mg/kg, 130 mg/kg, 260 mg/kg, and 520 mg/kg). At the same time, the long-term administration group was also subdivided into the blank control group, model group, and administration group (65 mg/kg and 520 mg/kg). The animals in the model and administration groups were allowed to feed freely in a single case and subjected to chronic unpredictable mild stress (CUMS) program to make the model. In contrast, the blank control group was fed in cages without subjecting to CUMS for 56 days. The institutional ethical review board approved the study protocol before starting any experiments on animals.

Following model development in the administration group, the animals were administered Shuganjieyu capsules solution at dosages of 65 mg/kg, 130 mg/kg, 260 mg/kg, and 520 mg/kg, respectively. The blank and model groups were treated with the same amount of water twice a day for one day and then fasted.

### 2.3. Development of CUMS Depression Model

CUMS program stimulation factors include the following [7]: overnight lighting, fasting, water banning, hot water swimming, and cold water swimming. The above stimulation factors were randomly assigned seven days a week, and two kinds of compound factor stimulation were randomly arranged daily.

The rat depression model was evaluated by measuring the rat body weight [8], rat sugar water preference [9], and rat immobility time [10].

### 2.4. Extraction of Liver Microsomes and Determination of Protein Concentration

The preparation of rat liver microsomes and the determination of protein content were done following the method reported earlier [11].

### 2.5. Liver Microsome Incubation

The total volume of liver microsome incubation system was 200 *μ*L, including 0.8 mg/mL liver microsomes, specific Cocktail probe substrate of each subenzyme (phenacetin 18 *μ*M, tolbutamide 18 *μ*M, dextromethorphan 20 *μ*M, omeprazole 12 *μ*M, and testosterone 80 *μ*M), with an added phosphoric acid buffer (0.1 mol/L, pH = 7.4) to make up the system to 180 *μ*L. The system was preincubated for 10 min in a water bath maintained at 37°C, followed by the addition of 20 *μ*L of NADPH. The mixture was again preincubated for 10 min at the same time to start the reaction and further incubated at 37°C in a water bath for 90 min. Following that, a total of 200 *μ*L of an internal standard containing 0.4 *μ*M cold terminator of dexamethasone was added to terminate the reaction, and the mixture was then vortexed at 18000 × g.

The chromatographic conditions for establishing the metabolite analysis method comprised phase A as an aqueous solution containing 0.1% formic acid and phase B comprised acetonitrile solution containing 0.1% formic acid. The mobile phase flow rate was adjusted to 0.2 mL/min. The optimal elution conditions were as follows: 0-2.2 minutes, 20-21% B; 2.2-8.5 minutes, 21-90% B; 8.5-9 minutes, 90-92% B; 9-9.3 minutes, 92% B; 9.3-9.6 minutes, 92-20% B; and 9.6-11.5 minutes, 20% B.

Mass spectrometric conditions for establishing analytical methods for metabolites comprised of positive ion mode for data collection. The mass scanning range was set at 100~1000 m/z, with a drying air flow rate of 9 L/min. The temperature of dry gas was fixed at 350°C, and 150 V was used as fragmentation voltage. Before measuring the sample, the calibration solution was used to calibrate the mass axis, and the mass accuracy error was adjusted to be less than 10 ppm.

### 2.6. Immunohistochemical Detection

Paraffin sections of the liver tissue were stained with microwave repair antigen, slightly counterstained with hematoxylin, dehydrated, transparent, neutral gum sealing, and examined under a microscope. The micro camera system was used to collect the images of the slices; the average optical density of the collected images was measured by Image-Pro Plus image analysis software.

### 2.7. Detection of mRNA Expression by RT-qPCR

Trizol reagent was used to extract total RNA from tissues as per instructions provided by the manufacturer. Reverse transcription synthesis of cDNA was done with Goldenstar™ DNA Synthesis SuperMix reagent, with GAPDH as an internal reference. The PCR product was amplified with EvaGreen 2X qPCR MasterMix kit after adding the primer of the target gene as given in Table 1.

## 3. Statistical Treatment

SPSS 16.0 statistical software was used. Measurement data were expressed by *x* ± *s*, and a *t*-test was used for comparison between groups. The difference was statistically significant when *P* < 0.05.

## 4. Result

### 4.1. Experimental Results of Single Administration Subgroup

#### 4.1.1. Establishment of CUMS Depression Model and Behavioral Evaluation after Administration

There were significant differences in body weight, sugar water preference, and immobility time between the model group, the administration group, and the blank group, indicating that the CUMS model was successful. The results are shown in Tables 2–4.

#### 4.1.2. Liver Microsome Incubation

It can be seen from Figure 1 that the conversion rates of CYP1A2 and CYP2C19 in the model group and the administration group were significantly higher than those in the blank group. The metabolic conversion rates of other enzymes did not change significantly, indicating that chronic unpredictable stimulation could induce CYP1A2 and CYP2C19 in rats and had no significant effect on CYP2D6, CYP3A4/5, and CYP2C9. A single dose of the Shuganjieyu capsule did not affect the activities of P450 enzymes.

#### 4.1.3. Immunohistochemical Detection

It can be seen from Figure 2 that the protein expression of CYP1A2 and CYP2C19 in the model group and the administration group was significantly higher than that in the blank group. The metabolic conversion rates of other enzymes were not significantly changed, indicating that chronic unpredictable stimulation could promote the protein expression of CYP1A2 and CYP2C19 in rats and had no noticeable effect on CYP2D6, CYP3A4/5, and CYP2C9. A single dose of the Shuganjieyu capsule did not affect the protein expression of P450 enzymes.

### 4.2. Experimental Results of Long-Term Administration Subgroup

#### 4.2.1. Establishment of CUMS Depression Model and Behavioral Evaluation after Administration

The results showed that the body weight and sugar water preference of CUMS rats were significantly lower than those of blank rats, and the immobility time of CUMS rats was significantly higher than that of blank rats. After three months of the administration, the body weight and sugar water preference of rats in the administration group were significantly higher than those in the model group. It shows that the Shuganjieyu capsule can treat the behavioral effects of chronic unpredictable stimuli on rats. (Tables 5–7).

#### 4.2.2. Liver Microsome Incubation

It can be seen from Figure 3 that the conversion rates of CYP1A2 and CYP2C19 in the model group were significantly higher than those in the blank group. The increase could be reversed in the administration group, and the metabolic conversion rates of other enzymes did not change significantly. The results showed that the Shuganjieyu capsule could inhibit the increase of liver CYP1A2 and CYP2C19 activities induced by the CUMS model in rats.

#### 4.2.3. Immunohistochemical Detection

It can be seen from Figure 4 that the protein expression of CYP1A2 and CYP2C19 in the model group was significantly higher than that in the blank group, and the increase could be reversed in the Shuganjieyu capsule group, while the expression of other enzymes was not significantly changed. The results showed that the Shuganjieyu capsule could inhibit the increase of CYP1A2 and CYP2C19 protein expression in a rat liver induced by the CUMS model.

## 5. Discussion

In this study, the depression model rats induced by CUMS program were used as the research object, and the Shuganjieyu capsule was used for treatment. The results show that the Shuganjieyu capsule can effectively improve the depressive symptoms of CUMS depression model rats. Some studies have shown that its mechanism may be related to inhibiting a large amount of extracellular Ca2+ influx, preventing Ca2+ overload, and downregulating the expression of the caspase-3 protein in the brain [12].

Since Chinese patent medicine can induce or inhibit CYP450 activity after the observation period, we used liquid chromatography-mass spectrometry (LC-MS) based on the Cocktail probe substrate method to explore the effect of Shuganjieyu capsule on CYP450 enzyme. The constructed Cocktail probe substrate method and mouse liver microsome coincubation method can simultaneously detect the inhibitory effect of the tested substance on five CYP450 enzyme subtypes at high speed. Compared with the higher conversion rates of CYP1A2 and CYP2C19 in the model group, the administration group of the Shuganjieyu capsule can inhibit the increase of liver microsomal CYP1A2 and CYP2C19 activities in CUMS depression rats. In addition, long-term administration of Shuganjieyu capsule can downregulate the activities of CYP1A2 and CYP2C19 enzymes in CUMS depression model rats by inhibiting the expression of CYP1A2 and CYP2C19 proteins and CYP1A2 mRNA, indicating that the metabolism of Shuganjieyu capsule in the liver is mainly through two CYP450 enzyme subtypes of CYP1A2 and CYP2C19, and may affect the bioavailability of drugs metabolized by CYP1A2 and CYP2C19 enzymes. It is suggested that in the clinical application of the Shuganjieyu capsule combined with other drugs through CYP1A2 and CYP2C19 metabolic pathways, attention should be paid to, and the dosage should be adjusted if necessary.

In conclusion, this study evaluated the effect of the Shuganjieyu capsule on CYP450 enzyme activity in treating depression and guided clinical development and application. In the following experimental research work, we will devote ourselves to using high-resolution and high-sensitivity analysis technology to study the action mechanism of a single drug and single drug of Shuganjieyu capsule, further explore the effect and quantitative degree of Shuganjieyu capsule on CYP450 enzyme subtype, and provide guidance for later clinical medication.

## Figures and Tables

**Figure 1:** The conversion rate of P450 Enzyme in the single-dose subgroup. Compared with the blank group, ∗∗ means *P* < 0.01.

**Figure 2:** Immunohistochemical assay in the single-dose subgroup. Compared with the blank group, ∗∗ means *P* < 0.01.

**Figure 3:** The conversion rate of the P450 Enzyme in the multiple-dose subgroup. Compared with the blank group, ∗∗ means *P* < 0.01. Compared with the model group, ## means *P* < 0.01.

**Figure 4:** Immunohistochemical assay in the multiple-dose subgroup. Compared with the blank group, ∗∗ means *P* < 0.01. Compared with the model group, ## means *P* < 0.01.

**Table 1:** The primer sequences.

Gene name	Primer sequence (5′-3′)
CYP1A2	F: GTCACCTCAGGGAATGCTGTG R: GTTGACAATCTTCTCCTGAGG
CYP2C9	F: CTGCTGCTGCTGAAACACG R: TTTCATGCAGGGGCTCCG
CYP2C19	F: TGGTCCACGAGGTTCAGAGATACA R: GGTTGGGAAACTCCTTGCTGTCAT
CYP2D6	F: TGCGAGAGGCACTGGTGA R: CGTGGTCCAAAGCCCGAC
CYP3A5	F: GGCAAACCTGTCCCTGTGAAAGA R: CTGGCGTGAGGAATGGAAAGAGT
CYP3A4	F: GGCAAACCTGTCCCTGTGAAAGA R: CTGGCGTGAGGAATGGAAAGAGT
GAPDH	F: TGCTGAGTATGTCGTGGAG R: GTCTTCTGAGTGGCAGTGAT

**Table 2:** Effect of CUMS model on rat body weight (*n* = 6).

Group	Dose (mg/kg)	Weight before modeling (g)	Modeling 56-day body weight (g)
Blank group	—	189.5 ± 6.19	410.67 ± 15.23
Model group	—	190.67 ± 4.84	318.5 ± 8.41^∗∗^
Administration group	65	187.17 ± 2.99	322.33 ± 12.21^∗∗^
	130	193.17 ± 6.37	323.33 ± 4.49^∗∗^
	260	193.33 ± 5.99	321.83 ± 19.72^∗∗^
	520	189.33 ± 1.21	329.5 ± 8.6^∗∗^

Compared with the blank group, ∗∗ means *P* < 0.01.

**Table 3:** Effect of CMUS model on sucrose preference test (*n* = 6).

Group	Dose (mg/kg)	Sugar water preference before modeling (%)	Modeling 56-day sugar water preference (%)
Blank group	—	78.14 ± 11.24	81.92 ± 8.43
Model group	—	80.27 ± 8.86	50.28 ± 19.51^∗^
Administration group	65	78.85 ± 9.83	43.87 ± 27.92^∗∗^
	130	81.46 ± 8.98	56.03 ± 18.36^∗^
	260	76.76 ± 9.96	42.3 ± 21.19^∗∗^
	520	77.74 ± 9.59	46.55 ± 24.24^∗∗^

Compared with the blank group, ∗ means *P* < 0.05 and ∗∗ means *P* < 0.01.

**Table 4:** Effect of CUMS model on forced swim test (*n* = 6).

Group	Dose (mg/kg)	Swimming immobility time (S)
Blank group	—	3.67 ± 1.86
Model group	—	65.33 ± 21.4^∗∗^
Administration group	65	63.5 ± 31.85^∗∗^
	130	65.17 ± 29.04^∗∗^
	260	65.17 ± 21.55^∗∗^
	520	54.17 ± 10.09^∗∗^

Compared with the blank group, ∗∗ means *P* < 0.01.

**Table 5:** Effect of CUMS model on rat body weight (*n* = 6).

Group	Dose (mg/kg)	Weight before modeling (g)	Body weight on 56th day of modeling (g)	Body weight after three months of administration (g)
Blank group	—	212.22 ± 4.57	465.75 ± 13.78	488.17 ± 21.97.
Model group	—	214.48 ± 9.53	334.02 ± 20.41^∗∗^	377.83 ± 22.94^∗∗^
Administration group	65	212.12 ± 7.62	328.17 ± 27.89^∗∗^	486.47 ± 24.06^##^
	520	215.17 ± 6.97	325.2 ± 26.31^∗∗^	485.67 ± 22.83^##^

Compared with the blank group, ∗∗ means *P* < 0.01. Compared with the model group, ## means *P* < 0.01.

**Table 6:** Effect of CMUS model on sucrose preference test (*n* = 6).

Group	Dose (mg/kg)	Sugar water preference before modeling (%)	Sugar water preference after 56 days of modeling (%)	Sugar water preference after three months of administration (%)
Blank group	—	82.41 ± 7.03	82.56 ± 7.45	84.25 ± 7.47
Model group	—	84.36 ± 6.77	54.91 ± 8.81^∗∗^	56.97 ± 8.71^∗∗^
Administration group	65	83.37 ± 9.95	50.48 ± 14.85^∗∗^	84.6 ± 7.75^##^
	520	80.43 ± 7.75	53.09 ± 10.43^∗∗^	84.35 ± 6.4^##^

Compared with the blank group, ∗∗ means *P* < 0.01. Compared with the model group, ## means *P* < 0.01.

**Table 7:** Effect of CUMS model on forced swim test (*n* = 6).

Group	Dose (mg/kg)	56-day swimming immobility time for modeling (S)	Swimming immobility time for three months after administration (S)
Blank group	—	12.67 ± 5.61	9.5 ± 3.83
Model group	—	45 ± 29.4^∗∗^	45 ± 16.12^∗∗^
Administration group	65	41.83 ± 17.5^∗∗^	11.17 ± 4.71^##^
	520	40.67 ± 17.19^∗∗^	10.67 ± 4.08^##^

Compared with the blank group, ∗∗ means *P* < 0.01. Compared with the model group, ## means *P* < 0.01.

## Data Availability

All the data about this paper is presented in the paper. If further information is required, a proper request shall be addressed to the corresponding author.
